The article "A Multimodel Fusion Method for Cardiovascular Disease Detection Using ECG" was retracted in 2023. Reasons: signs of a paper mill; compromised peer review; unreliable results or conclusions.

# A Multimodel Fusion Method for Cardiovascular Disease Detection Using ECG

**DOI:** 10.1155/2022/3561147

**Published:** 2022-05-16

**Authors:** Guanghui Song, Jiajian Zhang, Dandan Mao, Genlang Chen, Chaoyi Pang

**Affiliations:** ^1^School of Computer and Data Engineering, Ningbo Tech University, Ningbo 315100, Zhejiang, China; ^2^Department of Electrocardiogram, Ningbo Hospital of Traditional Chinese Medicine, Ningbo 315100, Zhejiang, China

## Abstract

*Objective*. Electrocardiogram (ECG) is an important diagnostic tool that has been the subject of much research in recent years. Owing to a lack of well-labeled ECG record databases, most of this work has focused on heartbeat arrhythmia detection based on ECG signal quality. *Approach.* A record quality filter was designed to judge ECG signal quality, and a random forest method, a multilayer perceptron, and a residual neural network (RESNET)-based convolutional neural network were implemented to provide baselines for ECG record classification according to three different principles. A new multimodel method was constructed by fusing the random forest and RESNET approaches. *Main Results.* Owing to its ability to combine discriminative human-crafted features with RESNET deep features, the proposed new method showed over 88% classification accuracy and yielded the best results in comparison with alternative methods. *Significance*. A new multimodel fusion method was presented for abnormal cardiovascular detection based on ECG data. The experimental results show that separable convolution and multiscale convolution are vital for ECG record classification and are effective for use with one-dimensional ECG sequences.

## 1. Introduction

The electrocardiogram (ECG), which reflects the heart's electrical activities, is widely used in clinics and hospitals worldwide to diagnose cardiac disorders. According to Bacquera et al. [1], the ECG signal itself is effective for predicting many cardiovascular-related diseases. However, because of the complexity and variability of ECG signals, it takes years to train a professional cardiologist to interpret them. Furthermore, the growing number of people with cardiac diseases makes the situation worse.

Therefore, an automatic and accurate system is needed to help doctors with ECG-based diagnoses. An ECG signal consists of five main waves, namely, *P*, *Q*, *R*, *S*, and *T*. Automatic classification systems can use the information hidden in ECG signals to assess heart-related diseases (e.g., atrial fibrillation), as different disorders result in different signal morphologies in both time and frequency domains. Thus, after the important features have been detected and a huge amount of data collected, it should be possible to automatically distinguish many heart-related diseases. As there are many types of heart-related disease, the first stage of ECG-based automatic diagnosis is to distinguish abnormal ECG signals from normal records. Then, cardiologists can concentrate on the signals that may reflect disease. More importantly, when used as an auxiliary diagnostic tool, such an automatic diagnosis algorithm could greatly reduce misdiagnosis rates. Thus, in this article, a binary ECG signal classification framework is presented and shown to achieve state-of-the-art results.

The article "A Multimodel Fusion Method for Cardiovascular Disease Detection Using ECG" was retracted in 2023. Reasons: signs of a paper mill; compromised peer review; unreliable results or conclusions.

In recent years, most ECG classification research has fallen into two categories: ECG heartbeat classification and lead classification. The heartbeat is the basic component of an ECG record. Luz et al. [2] surveyed the latest techniques for the detection of abnormalities based on ECG heartbeat classification. The algorithms involved in ECG lead classification are similar to those used for heartbeat discrimination.

### 1.1. Signal Preprocessing

Normally, three steps are performed to identify the label of an ECG record: (i) signal preprocessing, (ii) feature extraction and analysis, and (iii) signal classification. Preprocessing of signals normally consists of making a judgment regarding the noise level of an ECG signal and denoising the signal. Clifford et al. [3] proposed six signal quality indices to evaluate the quality of 12-lead ECG signals in the PhysioNet/Computing in Cardiology Challenge 2011 [4] and achieved good results for classifying the signals as acceptable or unacceptable. Empirical mode decomposition (EMD) and discrete wavelet transform (DWT) were used by [5] to denoise ECG signals.

### 1.2. Feature Extraction

Features extracted from signals are vital for the final classification task because the obtained feature vector is used as the representation of a record. Features in either the time domain or in the frequency domain were used. A combination of ECG signal morphological and dynamic features was used by Ye et al. [6] to classify heartbeats from the MIT-BIH arrhythmia database. Sarkaleh et al. [7] used DWT to extract features and formed a feature vector, which was used by a multilayer perceptron (MLP) to classify heartbeats. DWT is the most popular method used to extract features from the frequency domain [8–10]. EMD has also been used as an effective tool to extract features [11]. Given the complexity of ECG features and the powerful capabilities of deep learning, neural networks have been employed as feature extractors. Kiranyaz et al. [12] realized a real-time ECG classification system based on a one-dimensional (1-D) convolutional neural network (CNN) in which feature extraction and classification were both performed by the CNN model. Kachuee et al. [13] implemented a 13-weighted-layer network to extract features from ECG signals and learn representations of the signals. They trained the network for arrhythmia detection and successfully used their model to diagnose myocardial infarction.

The article "A Multimodel Fusion Method for Cardiovascular Disease Detection Using ECG" was retracted in 2023. Reasons: signs of a paper mill; compromised peer review; unreliable results or conclusions.

### 1.3. Classification Algorithms

After feature extraction, the formed feature vectors are fed into classifiers to obtain the final result. Over the past 20 years, a huge amount of work has been done on using machine learning and deep learning methods to classify ECG signals. The support vector machine (SVM) with kernel function is a popular method for classifying ECG signals [6, 14–16]. The random forest method is also widely used because of its simplicity and high classification accuracy [17–19]. As this method uses few parameters, it can achieve relatively good results without any tuning process. Based on its excellent performance in image classification tasks, deep learning is also used to classify ECG signals [8–11]. Furthermore, Moavenian et al. [16] performed a comparison between an SVM and an artificial neural network for classifying ECG signals. Their results showed that the SVM was more time-efficient, whereas the MLP had stronger generalization capability.

### 1.4. Record Classification

In addition to heartbeat classification, ECG signals can be classified based on the whole lead. The PhysioNet/Computing in Cardiology Challenge 2017 [20] aimed to classify ECG records into four classes based on a single ECG lead. Teijeiro et al. [21] used clinically meaningful features to train two classifiers, XGBoost and a long short-term memory network, to evaluate records globally and as a sequence. The outputs of the two classifiers were then combined to give the prediction result. Zabihi et al. [19] suggested a random forest model using features from time and frequency domains and phase space reconstruction; this model achieved high F1 scores. Hong et al. [22] extracted expert features and deep features (features extracted by a deep neural network) for classification. A cascaded binary classifier was implemented by Datta et al. [23] and proved to be very useful for record classification tasks. Normal and abnormal records differ from each other greatly, as shown in Figure 1. It is obvious from the figure that the abnormal ECG record has a much shorter R-R interval than the normal one.

Huang et al. [24] classified ECG signals from the Physikalisch-Technische Bundesanstalt database as normal or abnormal using three classifiers: stepwise discriminant analysis, SVM, and LASSO logistic regression. Zhang et al. [25] built the Chinese Cardiovascular Disease Database (CCDD), containing more than 100,000 12-lead ECG signals with well-labeled clinical diagnosis results, enabling classification of large-scale ECG records. Jin et al. [26] compared four traditional CNNs with a lead CNN (LCNN) in which they designed specifically for multilead ECG signals. The LCNN achieved the best results, with an 83.66% classification accuracy for distinguishing abnormal and normal ECG records. They then integrated two LCNNs and four rule-based classifiers; this combination yielded an accuracy of 86.22%. A Bayesian fusion method was used to combine two LCNN outputs; then, a Bayesian averaging method was applied to combine the results of the LCNN model and the rule-based classifiers and generate the final prediction [27]. Chen et al. [28] proposed a multibranch convolutional and residual network (MBCRNet), which had an average accuracy of 87.04%. Three feature fusion methods will be discussed in this paper.

The article "A Multimodel Fusion Method for Cardiovascular Disease Detection Using ECG" was retracted in 2023. Reasons: signs of a paper mill; compromised peer review; unreliable results or conclusions.

On the basis of previous work, we find that different methods produce different advantages in ECG classification tasks. Most of the work has focused on heartbeat classification; there have been fewer studies of classification based on whole ECG records. Therefore, in this work, we focused on distinguishing abnormal ECG signals based on whole 12-lead records. We proposed and compared three classification frameworks based on traditional machine learning, a 1-D residual neural network (RESNET), and a 2-D RESNET. CCDD was chosen as our experimental dataset. We achieved state-of-the-art performance in the normal/abnormal classification task based on CCDD ECG records.

The main contributions of our proposed method are as follows:

- We used both a signal quality filter and a record quality filter (RQF) to examine heavily polluted ECG records.
- We proposed a feature fusion method combining both local and global features of ECG signals to form a record feature vector.
- We analyzed the influence of multiscale convolution and separable convolution on multilead ECG records.
- We implemented three classification baselines and applied model fusion to obtain RF-MLP (random forest fused with MLP) and RF-RESNET (random forest fused with RESNET) models. Better classification results were achieved with the RF-RESNET model. To the best of our knowledge, this is the highest accuracy achieved for record classification work on the CCDD database.

This paper is organized as follows.  Section 1 summarizes related work on traditional and recently developed techniques applied to ECG diagnosis. In Section 2, we introduce the method and framework of our work. Detailed experiments and a discussion are presented in Section 3. Finally, we draw conclusions about our work in Section 4.

The article "A Multimodel Fusion Method for Cardiovascular Disease Detection Using ECG" was retracted in 2023. Reasons: signs of a paper mill; compromised peer review; unreliable results or conclusions.

## 2. Method

### 2.1. Dataset and Preprocessing

We obtained approximately 140,000 records from CCDD, labeled as normal or abnormal with respect to least one type of disease. As in [26], we further relabeled the data as normal (0) or abnormal (1) for binary classification based on the original labels. In detail, records with labels of “0 × 0101” or “0 × 020101” were relabeled as normal (0); the others are relabeled as abnormal (1). A Butterworth filter (Bfilter) was used to remove noise such as baseline wander. Raw ECG signals from 12 channels are fed into the Bfilter, and the denoised ECG signal is output. The default parameters of the Bfilter were set to order = 4, type = “lowpass.”

Records of less than 8 s in length and those mixed with too much noise were excluded using our proposed RQF algorithm, which will be described later. The original sampling rate was 500 Hz; for computational efficiency, we downsampled the signal to 200 Hz.

### 2.2. Record Quality Filtering

After applying various denoising methods, there were still some records that needed to be removed, as shown in Figure 2. These seriously damaged records were not suitable for use in classification work, as such noisy data do not retain the original pattern of real data and could cause the model to learn irrelevant features for the corresponding data type. Thus, based on the work of Orphanidou et al. [29], we developed our RQF, a fast feature-based ECG signal quality filter (Figure 3).

As shown in Figure 3, the first step was to detect *R* peaks and locate all the heartbeats in a record. Then, four rules were defined to set a threshold for unusable records. Here, HR is the heart rate, and max(|*RR*|) and min(|*RR*|) represent the maximum and minimum *R*-*R* intervals throughout the records, respectively. A feasible record should satisfy the following four conditions: HR less than 180 and more than 20; max(|*RR*|) not exceeding 3 s; the ratio of max(|*RR*|) to min(|*RR*|) less than 4; and, finally, number of *R* peaks more than 5 if a record is longer than 8 s.

Notably, our RQF does not need information about the QRS complex, *P* wave, or *T* wave; it only needs to identify all the *R* peaks in each record. The detection of an *R* peak yields the highest accuracy, as suggested by many studies.

Thus, our method also reduces the quality identification error originating from the wave delineation process. Through this filter, 1603 noisy records were removed from the dataset. Finally, we obtained 81,000 normal and 58,000 abnormal records for use as training and testing data, respectively.

The article "A Multimodel Fusion Method for Cardiovascular Disease Detection Using ECG" was retracted in 2023. Reasons: signs of a paper mill; compromised peer review; unreliable results or conclusions.

### 2.3. Feature Fusion

Representative features are vital for distinguishing one type of record from others. An ECG record can be represented as signal = {*L*^1^, *L*^2^, ..., *L*^*j*^}, where *j* represents the number of leads. In this work, *j* is equal to 12, and *L*^*i*^ is the ith-lead, L^i^ = {*a*_1_, *a*_2_,…, *a*_*n*_}, where *a*_*n*_ represents the voltage value at time step *n*. The heartbeat is the basic component of ECG records, and the relationship between heartbeats in the same or different leads contains dynamic information on heart activities. As the shape forms of a time interval at different leads reflect heart activities from different angles, abnormal patterns may present differently in different leads.

We, therefore, present a novel feature fusion method combining local and global features from 12 leads to form discriminative feature representations of ECG records.

- Local features are the features obtained from each heartbeat. For each heartbeat, features from the time and frequency domains and the wave morphology are calculated and combined to form a local vector, which represents the heartbeat.
- Global features consist of features computed from the whole ECG lead, namely, the R-R interval and DWT coefficients.

We implemented a modified QRS detection algorithm based on Pan et al. [30] to identify the *R* peak of each beat. We calculated the maximum amplitude, minimum amplitude, mean amplitude, and variation in amplitude for the obtained beats to describe the beat morphology. Based on [31], kurtosis signal quality indices were chosen to represent differences between the normal distribution and heartbeat data. We used skewness signal quality indices to measure the symmetry of a beat. A fast Fourier transform was performed on each beat to compute the wave energy (amplitude) and the frequency offset (phase). Fourth-order DWT coefficients were also used as features in the frequency domain. Based on our prior work [32], ten local features were chosen and are run on each of the 12 leads separately.

Global features are extracted from the lead scale. The *R*-*R* interval represents the heart rate variability, that is, the dynamic rhythm of the signal. We extract *R*-*R* intervals and their first-order differences. DWT is performed on the whole ECG lead, and sixth-order DWT coefficients are obtained as lead frequency features.

After local features and global features have been obtained, a two-stage feature fusion method is applied to form the final feature vector. First, for each lead, local and global features are combined to form the lead vector. Each lead is represented as a lead vector. Then, lead vectors are concatenated to form a record vector, *r* vector. The ECG record is represented as follows:

(1) $$\begin{array}{c} r\text{ vector}=\left[x_{i}^{\left(1\right)},x_{i}^{\left(2\right)},x_{i}^{\left(3\right)},\ldots ,x_{i}^{\left(P\right)}\right]\in R^{V\times P}, \end{array}$$

where *P* is the number of leads, *V* represents the volume of features in each lead vector, and *x*_*i*_^(*n*)^ represents the features of the *n*-th lead. In this work, *P*=12.

The article "A Multimodel Fusion Method for Cardiovascular Disease Detection Using ECG" was retracted in 2023. Reasons: signs of a paper mill; compromised peer review; unreliable results or conclusions.

### 2.4. Random Forest

Random forest is a traditional machine learning technique that shows powerful performance in many classification tasks. A random forest is constructed by building many decision trees based on bagging, and the final classification result is the average prediction or maximum vote of each decision tree. However, the random forest method does not simply combine the decision trees but randomly selects a subset of features at each split point, thereby overcoming the overfitting problem. When random selection is not used, decision trees tend to choose the most important feature set, resulting in high correlation among trees and low classification performance. One of the most important hyperparameters of the random forest method is the number of trees it builds for a given dataset. A grid search is used to determine the optimal number of trees for a record classification task. As described above, *re* vector={*x*_*i*_^1^, *x*_*i*_^2^, *x*_*i*_^3^,…, *x*_*i*_^*P*^} is the input feature vector. After training, for each *r* vector, the model outputs the probabilities for each record class. The class with the highest probability is regarded as the prediction label.

### 2.5. Multilayer Perceptron

MLP is the predecessor of CNN and consists of neurons and weights that connect neurons in different layers. In contrast to CNN, neurons in layer *L*_*i*_ in the MLP connect with all neurons in layer *L*_*i*−1_. Thus, information from the input vector can be preserved to the maximum extent in the network. For example, MLP architecture is shown in Figure 4.

Figure 4 shows a four-layer MLP. The first layer is the input layer receiving ECG feature vector {*x*_1_, *x*_2_, *x*_3_,…, *x*_*n*_}, where *n* is the length of the feature vector. Except for the bias neuron, each neuron receives one feature element *x*_*i*_. The last layer, which contains two neurons, is the output layer. The size of the output layer corresponds to the number of classes used for prediction. The two layers in between are hidden layers, mapping the input vector to the output classes through training and updating the weights of each perceptron. In our model, there are two hidden layers, each with 50 neurons, one input layer, and one output layer. The number of neurons in the input layer varies with the length of the feature vector extracted from the ECG record. The output layer contains two perceptrons, giving possible classes 0 and 1.

The article "A Multimodel Fusion Method for Cardiovascular Disease Detection Using ECG" was retracted in 2023. Reasons: signs of a paper mill; compromised peer review; unreliable results or conclusions.

### 2.6. Modified RESNET

Although deep representation is vital for distinguishing different classes of objects, traditional deep neural networks suffer from difficulty in training. RESNET [33] was proposed to solve this vanishing gradient problem by using shortcut connections in the residual block. The core idea of RESNET is to enable gradients to flow to earlier layers directly through these shortcut connections. In the case of long series of ECG signals, we assume that the use of deep architecture is the most effective way to extract ECG representational features. Therefore, in this work, a novel deep CNN was designed based on residual block architecture (Figure 5).

As shown in Figure 5, for each scale, a feature extractor with 16 RESNET blocks was implemented to form the feature map, where *Sep Conv* represents separable convolution and different downsampling scales result in ECG signals at different scales. The details are given below.

Similar to images, ECG signals contain features of different levels. Inspired by ContextNet [34], we implemented a multiscale extraction module in our CNN architecture to extract multilevel ECG features. Specifically, ECG pyramids are fed into the neural network to capture ECG signal information at different scales; this information is then concatenated to form a multiscale feature vector. ECG pyramids consist of ECG signals produced by different downsampling scales, enabling the calculation of feature maps with different receptive fields. Using a multiscale extraction method, both global dynamic information and local signal rhythm can be captured in the feature vector. We defined the original ECG signal as *raw*. Different downsampling scales produce signal fragments with distinct lengths, described as *clip*. The calculation of each clip is performed using the following formula:

(2) $$\begin{array}{c} M=\frac{N}{S},\\ \beta_{k}=\frac{1}{S}\sum_{i=S*k}^{S\times \left(K+1\right)-1}\alpha_{i}, \end{array}$$

where *N* is the length of the original signal; raw={*α*_1_, *α*_2_, *α*_3_,…, *α*_*n*_}, where 0 ≤ *i* ≤ *N*; *S* represents the downsampling scales {1, 2, 4, 8, 16}; and *M* is the length of the generated ECG clip. Therefore, the generated ECG pieces are clip={*β*_1_, *β*_2_, *β*_3_,…, *β*_*n*_}. Specifically, when *S* = 1, clip is the same as the original signal raw. Thus, with different values of S, multiClips is obtained as the new input signal series:

(3) $$\begin{array}{c} \text{multi Clips}=\left\{{\text{clip}}^{1},{\text{clip}}^{2},{\text{clip}}^{3},\ldots ,{\text{clip}}^{n}\right\}, \end{array}$$

where clip^*j*^ represents clip with a downsampling scale of *j*. To explore the effects of combinations of different downsampling scale clips, we performed experiments and discuss the results below.

The article "A Multimodel Fusion Method for Cardiovascular Disease Detection Using ECG" was retracted in 2023. Reasons: signs of a paper mill; compromised peer review; unreliable results or conclusions.

Considering ECG leads as channels in an image, 12 leads contain information from 12 channels. In clinical scenarios, different leads reflect various details of heart activity, and all leads are vital for judging the condition of the heart. Thus, all 12 channels were fed into the neural network for feature extraction. More importantly, although different leads have the same size, they are not exactly aligned. Along the dimension of time, the same heart activity causes the 12 leads to react slightly differently. Therefore, separable convolution was used in the convolution layers for better feature extraction. The first step is depth-wise convolution. Each channel is convolved by a kernel; different channels are computed separately. Suppose the number of channels is *C*, that is, *C* = 12. After depth-wise convolution, *C* feature maps are generated. The second convolution step fuses features from different channels by convolution in the depth dimension. This point-wise convolution combines features at similar spatial points across the *C* channels. Another significant advantage of separable convolution is the reduction of parameters in the neural network and of the overall model size. The training time is also shortened significantly. For comparison purposes, we implemented a modified RESNET based on CNN RESNET^c^ from [35] to classify normal and abnormal ECG records. Our model only contains 0.74 million parameters, whereas RESNET^c^ has more than 16 million; that is, it has 20 times fewer parameters.

After the feature extraction module, a fully connected layer is implemented to concatenate features. The fully connected layer is followed by a softmax layer, which is used as the classifier to predict the labels of ECG records.

### 2.7. RF-MLP

Random forest and MLP were trained separately using the r *vector* constructed in the feature fusion step. These two models were trained via different principles. When constructing decision trees, a random subset of features is selected at each split point. In our random forest model, decision trees are trained based on information gain theory. The MLP model trains the network through updating weights of neurons. Binary cross-entropy is used to calculate the loss in each iteration; then, backpropagation is applied to transfer the loss to previous layers for updating of weights. Therefore, the random forest and MLP methods have different training and classifying criteria. Proper fusion of these two models could enable better distinguishing ability.

The article "A Multimodel Fusion Method for Cardiovascular Disease Detection Using ECG" was retracted in 2023. Reasons: signs of a paper mill; compromised peer review; unreliable results or conclusions.

Random forest and MLP give probabilities for all prediction classes, where a high probability indicates a high confidence level. The class with the highest confidence level is defined as the prediction label. As mentioned above, because of the different characteristics of random forest and MLP, they may classify the same record into different classes. Thus, a probabilistic model fusion approach was implemented to make use of the advantages of both methods.

### 2.8. RF-RESNET

The main characteristic of our modified RESNET architecture is its ability to extract deep representations of ECG sequences. However, as it uses human-crafted features, *r* vector, random forest has stronger interpretability. As representatives of traditional machine learning algorithms and prevalent deep learning methods, the random forest and modified RESNET models could complement each other owing to their specific characteristics. The random forest model was trained with feature representation vector, *r* vector, whereas for the modified RESNET model, different ECG pyramids were used as training data. As in the case of random forest and MLP, a probabilistic model-fusion methodology was applied to make use of the advantages of the two models. During testing, the two models produced possibilities for each ECG instance, indicating the predicted class. Then, the model with the higher test accuracy was given greater weight in the final decision regarding the predicted class, and the architecture is shown in Figure 6.

## 3. Results and Discussion

Three independent normal/abnormal detection methods, random forest, MLP, and modified RESNET, were used as baselines. Two fusion models, RF-MLP and RF-RESNET, were evaluated with respect to their effectiveness in ECG record classification tasks. In total, five models were evaluated on the CCDD database to determine their ability to classify normal and abnormal ECG records.

The whole database was randomly partitioned into a training set, validation set, and test set using a ratio of 8 : 1 : 1. The validation set was used for early stopping and selection of hyperparameters for MLP and CNN. Then, models were evaluated on the test set to assess final performance.

For random forest evaluation, we set the parameter expressing the number of constructed trees to be 200, which has been demonstrated to be the best size for this work by a series of experiments.

The MLP used in this work consisted of four layers. Each hidden layer contained 50 neurons. *ReLU* and *sigmoid* were used as the activation functions of the hidden layer and the output layer, respectively. The MLP was trained with Adam, and *β*_1_ and *β*_2_ were set to 0.9 and 0.999, respectively. The input layer received record feature vectors as input data, and the output layer predicted the record classes.

The article "A Multimodel Fusion Method for Cardiovascular Disease Detection Using ECG" was retracted in 2023. Reasons: signs of a paper mill; compromised peer review; unreliable results or conclusions.

Our proposed CNN contains 34 layers. Before training the network, ECG sequences were intercepted to the same lengths. Then, *Z*-normalization was applied to the training, validation, and testing sets, respectively. Our RESNET-based CNN was trained with a ReLU activation function and Adam optimizer. The binary cross-entropy was used as the loss function. In each residual block, the convolution layer was followed by a dropout of 0.4. The final CNN contained 33 convolution layers and a fully connected layer. A sigmoid was applied to predict the two classes. The classification results obtained with these three models are shown in Table 1.

In Table 1, specificity is defined as the proportion of correctly predicted negative samples to the total number of samples with negative labels. Negative samples are those ECG records with abnormal behaviors. Therefore, a high specificity value means that most of the abnormal records were detected by the model. In this work, all three baseline models yielded specificity values of over 91%, which are vital in clinical applications.

Good results were achieved for ECG classification on the CCDD database, as listed in Table 2. Our models achieved high classification accuracy, and the fusion of random forest and modified RESNET yielded the best results. Furthermore, part of the PTB diagnostic ECG database, which contains 126 records of 12-lead ECGs from 43 patients, was also used for experiments, and the classification accuracy was 0.841 for our models.

We compared the difference in performance between separable and nonseparable convolution in CNN architecture. According to our experimental results, the classification accuracy was 0.831 for nonseparable convolution but 0.842 for separable convolution. Moreover, separable convolution required 20 times fewer parameters than nonseparable convolution. Therefore, for multichannel time-series data, separable convolution had a stronger distinguishing capability.

Furthermore, we conducted experiments using different convolutional scales to determine the influence of scale on the effectiveness of multiscale convolution methods. Details of the classification results are given in Figure 7. The modified RESNET achieved the best classification accuracy when the scale was 3. This implies that using too many scales leads to information redundancy. When the downsampling rate exceeds a certain level, key information in the original signal can become indistinguishable.

The article "A Multimodel Fusion Method for Cardiovascular Disease Detection Using ECG" was retracted in 2023. Reasons: signs of a paper mill; compromised peer review; unreliable results or conclusions.

To evaluate the effect of the depth of the modified RESNET, 34-layer and 50-layer modified RESNET models were implemented for comparison. The 50-layer network, which had 1.1 million parameters compared with 0.74 million in the 34-layer network, suffered from overfitting and had a training accuracy of approximately 0.9 and test accuracy less than 0.855.

## 4. Conclusion

In this work, we researched methods for the detection of normal/abnormal ECG signal records, which is the essential first step in ECG diagnosis. Owing to the presence of various types of noise in the ECG data, we proposed a record filtering method to remove records seriously affected by noise. Then, we developed a feature fusion method that could extract both local and global features from different leads to construct a representation of the ECG record. Random forest, MLP, and modified RESNET were implemented to provide classification baselines. Ensemble methods were developed by fusing random forest with MLP and RESNET, respectively. Experiments were performed to further investigate the influence of multiscale convolution and separable convolution. The best results were achieved when random forest was fused with modified RESNET, with three scales and separable convolution. The classification results for our methods were compared with those obtained with several state-of-the-art methods on the same database; our ensemble model using random forest and modified RESNET achieved the best classification results. Future work will include optimizing the algorithm and exploring the use of RNN and CNN models to enhance the accuracy of the method and its ability to extract dynamic features.

## Figures and Tables

**Figure 1:** Normal (*N*) and abnormal (*A*) records from CCDD.

**Figure 2:** Noisy records.

**Figure 3:** Record quality filter.

**Figure 4:** MLP architecture.

**Figure 5:** Modified RESNET architecture.

**Figure 6:** Model fusion architecture.

**Figure 7:** Classification results with different scales.

**Table 1:** Classification results for random forest, MLP, and modified RESNET.

Models	Precision	Recall	Specificity	F1 score	Accuracy
Random forest	0.888	0.795	0.928	0.839	0.872
MLP	0.861	0.733	0.915	0.792	0.839
Modified RESNET	0.869	0.762	0.920	0.812	0.855

**Table 2:** Summary of record classification performance on CCDD.

Literature	Method	Accuracy
Jin et al. [26]	LCNN	0.837
Jin et al. [27]	LCNNs and rule-based classifiers	0.862
Chen et al. [28]	MBCRNet-L	0.870
Proposed_1_	RF-MLP	0.874
Proposed_2_	RF-RESNET	0.880

## Data Availability

The data that support the findings of this study are available from the corresponding author upon reasonable request.
